This article has been retracted.

# Analysis of Predictive Model of Coronary Vulnerable Plaque under Hemodynamic Numerical Simulation

**DOI:** 10.1155/2022/3434910

**Published:** 2022-01-07

**Authors:** Qiang Song, Mingwei Chen, Jin Shang, Zhi Hu, Hui Cai

**Affiliations:** ^1^Department of Structural Heart Disease, The First Affiliated Hospital of Xi'an Jiaotong University, Xi'an 710061, China; ^2^Department of Respiratory and Critical Care Medicine, the First Affiliated Hospital of Xi'an Jiaotong University, Xi'an 710061, China; ^3^Department of Medical Iimaging, the First Affiliated Hospital of Xi'an Jiaotong University, Xi'an 710061, China; ^4^Department of Vascular Surgery, the First Affiliated Hospital of Xi'an Jiaotong University, Xi'an 710061, China

## Abstract

**Objective:**

Vulnerable plaque is considered to be the cause of most clinical coronary arteries, and linear cytokines are an important factor causing plaque instability. Early prediction of vulnerable plaque is of great significance in the treatment of cardiovascular diseases.

**Methods:**

Computational fluid dynamics (CFD) was used to simulate the hemodynamics around plaques, and the serum biochemical markers in 224 patients with low-risk acute coronary syndrome (ACS) were analyzed. Vulnerable plaques were predicted according to the distribution of biochemical markers in serum.

**Results:**

CFD can accurately capture the hemodynamic characteristics around the plaque. The patient's age, history of hyperlipidemia, apolipoprotein B (apoB), adiponectin (ADP), and sE-Selection were risk factors for vulnerable plaque. Area under curve (AUC) values corresponding to the five biochemical markers were 0.601, 0.523, 0.562, 0.519, 0.539, and the AUC value after the combination of the five indicators was 0.826.

**Conclusion:**

The combination of multiple biochemical markers to predict vulnerable plaque was of high diagnostic value, and this method was convenient and noninvasive, which was worthy of clinical promotion.

## 1. Introduction

Cardiovascular disease has become the leading cause of death worldwide. In China, cardiovascular diseases account for about half of the deaths caused by diseases and have become the number one cause of death in China. Every year, many patients cause great pressure on medical institutions, which causes great burden to the country and the people [1]. Coronary atherosclerotic heart disease, as a typical cardiovascular disease, is a chronic progressive inflammatory disease [2]. In terms of anatomical structure, arterial vessels are divided into the intima, media, and outer membrane from inside to outside. The intima, as the innermost layer of vascular wall, is the thinnest in structure and mainly composed of the endothelium and subendothelial layer [3]. The outer membrane is composed of loose connective tissue rich in elastic fibers and collagen fibers, which is responsible for supporting the vascular wall of the body [4]. The media is located between the intima and the outer membrane, and its composition and thickness vary with different blood vessel types in the human body [5]. Anatomically, the endothelial cells of the blood vessels in the intima are usually seen in direct contact with the blood. Therefore, it is mainly affected by the combined effect of the wall shear stress (WSS) of blood on the vascular wall and the peripheral circumferential stress (CS) of the solid [6, 7].

To date, many researchers focused on the mechanisms underlying the transition from chronic to acute coronary heart disease. Acute coronary syndromes (ACS) include unstable angina pectoris and ST-segment and non-ST-segment elevation acute myocardial infarction. More than half of the patients with ACS had no history and symptoms before onset [8, 9]. Based on massive cell, animal experiments, and clinical studies, it was found that the main cause of ACS is the formation of vulnerable plaques in patients' blood vessels and secondary acute vascular thromboembolism [10]. Therefore, the pathological basis of ACS includes vulnerable plaques, vulnerable myocardium, and vulnerable blood [11]. Vulnerable plaques include all plaques with rupture tendency or surface erosion, and rupture plaques are the main ones with complex causes. Some studies suggested that it may be due to the accumulation of blood-derived lipids in the lining of blood vessels and an immune reaction with white blood cells in the blood. After the reaction, the two cells entered the vascular endothelial cells and moved to the intima. After being cleaned by macrophages, lesions occurred in the vascular wall. Occlusive plaques and nonobstructive plaques are formed in the later stage of the disease, and the nonobstructive plaques rupture and form occlusive thrombus [12, 13].

The high occult nature of ACS leads to high morbidity and mortality of patients. Therefore, early identification and prediction of vulnerable plaques are of great significance for the diagnosis and treatment of ACS. At present, in addition to traditional computed tomography (CT) and magnetic resonance imaging (MRI), intravascular ultrasound (IVUS), optical coherence tomography (OCT), and coronary arteriograpphy (CAG) have also developed and appeared [14]. The aforementioned treatment methods can accurately identify vulnerable plaques and analyze plaque characteristics, but they all belong to invasive examination. In addition to the intolerances of some patients, it is also difficult to make accurate early diagnosis for dynamic changing vulnerable plaques. In addition to the shape and function of the plaque, the hemodynamic distribution of the plaque is also an important factor in determining whether the plaque ruptures or not [15]. Therefore, the study of plaque hemodynamic changes may be an important method for noninvasive diagnosis of ACS. The instability process of plaque from stable to unstable is the result of many factors. Inflammatory factors play a role throughout the development of the disease, and the development of the disease is not a linear process. During the period, it is affected and regulated by a variety of factors. The number of various factors in the blood is huge, and there are intricate influences among various factors. Therefore, combining multiple biochemical markers can more accurately and comprehensively reflect disease occurrence. It is of great significance to guide the diagnosis and treatment of subclinical coronary heart disease and reduce unnecessary radiation exposure and economic burden.

## 2. Materials and Methods

### 2.1. Hemodynamics of Vulnerable Plaques

From a fluid mechanical point of view, the body's cardiovascular system shows a wide range of flow phenomena. The blood is turbulent as it flows through the ascending aorta, which eddies as it flows through the aortic valve into the artery. When there is a large pressure gradient in blood, boundary-layer blood flow separation is easily caused by factors such as adverse pressure and viscosity [16]. These abnormal blood flow patterns may be related to the formation of vulnerable plaques.

At present, many studies confirmed that the occurrence of ACS is related to changes in inflammatory markers in the blood, and that inflammation is closely related to the instability of plaques. Therefore, inflammatory markers have great value in the diagnosis, treatment, and prognosis of ACS [17]. At present, common inflammatory-related biochemical markers include adiponectin (ADP), intercellular adhesion factor, selectin, integrin, immunoglobulin, myeloperoxidase (MPO), and matrix metalloproteinase (MMP). With adiponectin as an example, its role is secreting biologically active cytokines and hormones such as interleukin-6/8 and leukocyte chemotactic protein (MCP-(1)). These cytokines can regulate energy balance and hormone metabolism [18]. In the study of Kanaji et al. (2020) [19], it was found that patients with non-ST-segment elevation ACS undergoing percutaneous coronary intervention for one month were related to ADP and coronary artery blood flow reserve (g-CFR) impairment. In the g-CFR impaired group, there were remarkable differences in the location of the crime lesion, the level of amino-terminal B-type natriuretic peptide precursor, the level of high-sensitivity c-reactive protein (hs-CRP), and the ADP around the coronary arteries. A single-center retrospective study by Goeller et al. (2018) [20] also reported similar views. It was found that the low attenuation and intermediate attenuation of the crime plaque of ACS patients increased the NCP load. The correlation between CT attenuation and intermediate attenuation of ADP around the diseased coronary artery was strong.

The hemodynamics of ACS patients can also be evaluated by computational fluid dynamics (CFD) methods [21]. When the CFD method is adopted, it is necessary to solve the fluid dynamics control equation and then establish a hemodynamic model. In addition, the fluid mechanics problem is simulated and analyzed to capture the changes in the blood flow field before and after the plaque in ACS patients. The motion of the fluid should satisfy the continuity equation and the Navier-Stocks equation. A closed space in the fluid is taken and called a control volume. The surface of the control volume is called a control surface. According to the law of conservation of mass, after the fluid flows from the control surface h1 into the control body and then flows out from the control surface *h*2, the difference in mass is equal to the increase in the mass of the fluid in the control body. Based on this, the fluid fluidity equation can be obtained.

(1) $$\begin{array}{c} \frac{\partial }{\partial t}\underset{V}{∭}\rho \text{d}x\text{d}y\text{d}z+{∯}_{h}\rho \overset{⟶}{v}\cdot \overset{⟶}{n}dH=0. \end{array}$$

In equation (1), *V* represents the control body, *h* represents the control surface, (∂/∂*t*)∭_*V*_*ρ*d*x*d*y*d*z* represents the internal mass increase of *V*, and ${∯}_{h}\rho \overset{⟶}{v}\cdot \overset{⟶}{n}\text{d}H$ represents the net flux of *h* into *V*. According to the Ostrovski-Gauss formula, equation (1) is transformed into a differential form in a rectangular coordinate system, as shown below.

(2) $$\begin{array}{c} \frac{\partial \rho }{\partial t}+u\frac{\partial \left(\rho u\right)}{\partial x}+v\frac{\partial \left(\rho v\right)}{\partial y}+s\frac{\partial \left(\rho s\right)}{\partial z}=0. \end{array}$$

In equation (2), *ρ* represents the fluid density and (*u, v, s*) is the velocity at any point (*x, y, z*) in the flow field at time *t*.

For the vector form where the viscosity coefficient is constant and does not change with the coordinate position, the Navier-Stocks equation is expressed as the following equation:

(3) $$\begin{array}{c} \rho \frac{\text{d}\overset{⟶}{v}}{\text{d}t}=\rho \overset{⟶}{F}+\mu \nabla^{2}\overset{⟶}{v}-\text{grad}p+\frac{\mu }{3}\text{grad}\left(\text{div}\overset{⟶}{v}\right). \end{array}$$

For the vector form where the fluid density and viscosity coefficient are both constant conditions, the Navier-Stocks equation is expressed as the following equation:

(4) $$\begin{array}{c} \rho \frac{\text{d}\overset{⟶}{v}}{\text{d}t}=\rho \overset{⟶}{F}+\mu \nabla^{2}\overset{⟶}{v}-\text{grad }p. \end{array}$$

In equations (3) and (4), *ρ* represents the surface pressure and ∇ represents the Hamiltonian.

The purpose of the study on the pathological and physiological mechanisms of vulnerable plaques in ACS patients is conducting a more accurate quantitative analysis of the degree of ACS lesions to guide early clinical intervention to reduce the incidence and mortality of ACS. However, from the perspective of current studies, most of the current studies are focused on single biochemical markers with a small sample size. Multiple biochemical markers are expressed in various stages of plaque formation and development, interacted with each other, and are affected by systemic pathophysiological states. It is difficult for a single biochemical marker to accurately reflect the progression of plaque lesions and, therefore, is less representative. Based on this, this study was devoted to the construction of hemodynamic numerical models related to coronary artery vulnerable modules. A variety of biochemical indicators were combined and analyzed to provide more accurate information for the clinical prediction and prognosis of ACS (Figure 1).

### 2.2. Research Objects

In this study, 224 subjects who underwent CTA in our hospital from May 2020 to May 2021 were selected. All subjects were assessed by Framingham scoring system as low risk, and were rolled into experimental group (vulnerable plaque) with 102 cases and control group (nonvulnerable plaque, no plaque) with 122 cases according to the examination results. The baseline data of the two groups, including age, gender, smoking history, and family history, are shown in Table 1. This study had been approved by the ethics committee of the hospital. All subjects and their families had been informed about this study and signed informed consent.

### 2.3. Inclusion and Exclusion Criteria

Inclusion criteria: (i) age ≥18 years, gender was not limited; (ii) the participants were voluntary and had no symptoms related to coronary heart disease.

Exclusion criteria: (i) the patients were children and pregnant women; (ii) patients with congenital heart disease, cardiomyopathy, valvular disease, pericardium disease, and so on; (iii) patient who had a history of invasive heart surgery (including PCI, endovascular stenting, and heart bypass surgery); (iv) patient who had a history of diabetes and malignant tumor; (v) patients with systemic diseases that can lead to dyslipidemia; (vi) patient who was in the active stage of inflammatory lesions; (vii) patient who had pulmonary embolism; (viii) patient who had a recent history of trauma or surgery; (ix) patients who had various secondary hypertension, hyperthyroidism, blood system diseases, and so on.

### 2.4. CT CAG Method

CT scan was performed on all subjects in this study using Siemens Somatom definition DSCT scanner. The iodine allergy test was performed before scanning, and CT scan was performed after no adverse reactions were found. To avoid motion artifacts during the scan, the arrhythmias were taken orally 1 h before the scan. The patient underwent plain coronary artery scan followed by enhanced coronary artery scan. Collimator width was set to 128 × 0.614 mm, and tube voltage was 80–120 keV. The scan was made from the bifurcation to the bottom of the heart. A contrast agent was injected through the right elbow or wrist vein during the scan, using a double-barrel high-pressure syringe. The dosage of the contrast agent was 45–60 mL, and the injection flow rate was 5–6 mL/s. After the injection, 25 mL normal saline was injected at the same flow rate. The threshold value was set to 100–120 HU, the trigger layer was the root of the main artery, and the trigger delay time was set to 5 s.

### 2.5. Detection Methods

Four mL of fasting venous blood was extracted an hour before scanning, and serum was extracted by coagulation, centrifuged at 1,200 rpm for 10 min and stored at −80 °C. After the collection of all patients, the previously frozen serum was thawed and mixed by shaking and then diluted with FBS buffer at a dilution ratio of 1 : 350. Antibody cross-linking microspheres were prepared after dilution, and standard lines of quality control, lotion, serum matrix, and cytokine were prepared. In the ELISA test, 150 *μ*L reaction buffer was added to each well of the reaction plate, shaken at room temperature for 15 min, which was then filtered or discarded with absorbent paper. Then, 20 *μ*L reaction buffer was added to the sample wells, and 20 *μ*L standard and quality control were added to the corresponding wells; 20 *μ*L matrix solution was added to standard wells, quality control, and background, and 20 *μ*L samples were added to the sample well, oscillated at room temperature for 15 min. Then, 20 *μ*L mixed microspheres were added to each well. The plate was sealed and reacted at room temperature for two hours, then filtered, washed with 150 *μ*L PBS buffer solution twice, and dried with blotting paper. At room temperature, 20 *μ*L antibody was added to each well, and then 25 *μ*L Streptavicin-Rhycoerythrin was added to each well. After suction filtration, the plate was washed with 50 *μ*L PBS buffer solution twice, added with 150 *μ*L sheathing solution, oscillated for 10 min, and then read.

### 2.6. CFD-based Hemodynamic Model of Vulnerable Plaque

CFD is a method to simulate fluid movement in the blood flow field, which mainly simulates and analyzes some physical quantities in the variation of blood flow field, so as to subjectively present the distribution of some physical quantities such as velocity, momentum, and pressure [22]. The application of CFD is extremely wide. Wherever there is flow, CFD can be used for analysis. The numerical simulation of plaque blood flow consists of pretreatment, solution, and posttreatment.

The preprocessing stage divides the processing model into networks that computers can recognize and process. In this study, CT scan images of ACS patients were imported into ANSYS to establish the blood vessel model that could be recognized by the computer, and then the continuous governing equation was discretized, which required discretization of the computational region using partitioning networks, which divided the computational region into computable network forms. GAMBTI, ICEM CFD, and GRIDGEN are commonly used before dividing network. Taking GAMBTI preprocessor, as an example, can process mainstream computer aided design (CAD) data types and generate boundary layer networks, and it also has a good differentiation effect for complex geometry [23].

The solution phase mainly relies on FLUENT solver, including pressure-based solver and density-based solver. A pressure-based solver was selected, and pressure and momentum were taken as the main variables in data simulation. A typical pressure-velocity coupling algorithm, such as Coupled algorithm, updates the flow field variables first during calculation. The continuity, momentum, energy, and component equations are solved. Then, according to the governing equation, the auxiliary variable equations such as turbulence and radiation are solved until the equations converge.

Postprocessing refers to displaying the physical quantities obtained by the FLUENT solver. In this study, CFD-post software was used for CFD postprocessing.

### 2.7. Statistical Methods

Data in this study were processed with Excel 2019, and statistical analysis was performed with SPSS 22.0. Mean ± standard deviation ($\bar{x}$ ± *s*) was how measurement data were expressed, and percentage (%) was how count data were expressed. The *t*-test was used if the data were normal distribution, the rank-sum test was used if the data were not normal distribution, and the chi-square test was used for counting data. If multiple sets of data were compared with normal distribution, ANOVA was used. All the test results took *P* < 0.05 as statistically considerable difference.

## 3. Results and Discussion

### 3.1. Numerical Simulation Results of Hemodynamics around Plaque

In this study, a velocimetry platform was built to obtain images of microbubbles in plaques. The whole velocimetry platform was similar to a loop that like in Figure 2. It was composed of high-frequency ultrasonic imaging system, pulsation pump, and pressure transmitter. In addition, ultrasonic devices can obtain clear two-dimensional microbubble images. The high-frequency ultrasound imaging system detected the subject and produced a rectangular image. A pulsating pump was used to simulate the flow characteristics of human blood circulation system, and a pressure transmitter was responsible for regulating the fluid inlet and inlet pressure. During CFD simulation, the fluid pressure at the inlet and outlet can affect the simulation results. Therefore, a pressure transmitter was added for adjustment. The pressure transmitter can convert the pressure signal into electrical signal, which was convenient for oscilloscope acquisition. During the numerical simulation of hemodynamics, water was first added into the reservoir to generate pulsating flow by the pulsating pump. By adjusting pulsating pump frequency, stroke output, systolic/diastolic time ratio, and other parameters, the elastic blood vessel mimicked human blood vessels. Oscilloscopes, rotary flowmeters, and pressure sensors can measure experimental parameters. The contrast agent was injected into the circulation loop through the reservoir. The linear density, imaging depth, and imaging width of the ultrasonic imaging system were adjusted to obtain the best contrast image.

A high-frequency ultrasound imaging system was used to capture 1,200 frames of images (including 5 cardiac cycles), and then CFD was used to calculate the flow field. All images were selected as the velocity distribution images at the maximum cardiac cycle velocity (and the peak systolic period of the human body). In this study, the average velocities at the front, middle, and back three positions of the plaque under three degrees of stenosis of 30%, 50%, and 70% were studied. The simulated test results are shown in Figure 3.

### 3.2. Distribution Characteristics of General Biochemical Markers in Serum of Two Groups of Patients

General biochemical markers in the two groups were analyzed, including indicators related to glucose metabolism, lipid metabolism, cardiac function, and coagulation function. The distribution characteristics of general biochemical markers in the two groups are shown in Table 2.

### 3.3. Distribution of Special Biochemical Markers in Serum of Two Groups of Patients

Figure 4 presents the analysis of the distribution of seven special biochemical markers in the two groups of patients. The role of ADP was antiinflammatory and antiatherosclerosis. Soluble intercellular adhesion molecule (SICAM-1), E-selectin (sE-Selectin), P-selectin (sP-Selectin), MPO, and MCP-1 can promote inflammation and promote atherosclerosis. The ADP level of the control group was 8.61 ± 1.77, and that of the experimental group was 7.23 ± 1.54. The difference in ADP levels between the two groups was notable (*P* < 0.05). The experimental group's SICAM-1 (86.72 ± 22.15), sE-Selectin (72.11 ± 12.15), and MCP-1 (0.39 ± 0.08) were dramatically different versus the control group SICAM-1 (74.31 ± 20.18), sE-Selectin (61.39 ± 14.38), and MCP -1 (0.41 ± 0.09) (*P* < 0.05). These results also confirmed the antiinflammatory and antiatherosclerotic effects of ADP and the proinflammatory and atherogenic effects of SICAM-1, sE-Selectin, and MCP-1. However, no notable difference was observed between groups in SICAM-1, P-Selectin, and MPO (*P* > 0.05).

### 3.4. Prediction of the Occurrence of Vulnerable Coronary Plaques

The traditional risk factors of ACS and a variety of biochemical markers with *P* < 0.05 were used as dependent variables for Logistic regression analysis. The results showed that age, hyperlipidemia, apoB, ADP, and sE-Selectin were independent risk factors for vulnerable plaque. From this, the linear regression equation Logit *P* = −0.867 + 0.928 *x*_1_ + 0.709 *x*_2_ + 0.788 *x*_3_ - 0.831 *x*_4_ + 0.589 *x*_5_ was obtained, where *x*1 represented age, *x*2 represented hyperlipidemia, *x*3 represented apoB, *x*4 represented ADP, and *x*5 represented sE-Selectin. The ROC curve of the the five indicators on vulnerable plaques was plotted according to the linear regression equation, as shown in Figure 5.

According to the ROC curve of each index, the corresponding area under the curve was calculated, as shown in Figure 6. The results showed that the area under the curve (AUC) corresponding to age was 0.601, that corresponding to hyperlipidemia was 0.523, that corresponding to apoB was 0.562, that corresponding to ADP was 0.519, and that corresponding to sE-Selection was 0.539. However, it was one-sided to judge whether the factor was a risk factor for vulnerable plaques based solely on the area under the ROC curve corresponding to an independent variable. Therefore, the aforementioned five indicators were combined for judgment, and the AUC value obtained by combining the five variables was 0.826, which was greatly superior to the individual AUC value of any risk factor (*P* < 0.05). The results suggested that multiindex joint prediction had the best diagnostic effect on vulnerable plaques.

## 4. Conclusion

Vulnerable plaque is the pathological basis of ACS. In this work, it was found that CFD can accurately capture the hemodynamic characteristics around the plaque. As the degree of stenosis increased, the blood flow speed increased remarkably. For the ACS population with low and medium risk, a variety of serum biochemical markers were closely related to the occurrence of vulnerable plaques. Among them, age, hyperlipidemia, apoB, ADP, and sE-Selection were the risk factors for vulnerable plaque. Therefore, the clinic can predict vulnerable plaque by combining the aforementioned biochemical markers, with an AUC value of 0.826 and an ideal diagnostic effect. As a method of predicting intravascular hemodynamic distribution, CFD was applied to the prediction of vulnerable plaque for the first time in this study. Although the accuracy of CFD predicting vulnerable plaque required to be improved, this method was convenient, cheap, fast, and noninvasive and can provide clinical evidence for early clinical intervention and prognostic judgment of ACS patients. However, there are still some shortcomings in this study. The main blood biochemical table included is mainly related to inflammation and lipid metabolism. The impact of other related indicators on the occurrence of vulnerable plaques remains to be further studied.

## Figures and Tables

**Figure 1:** Image characteristics of different plaques. (a) No plaques; (b) calcified plaques; (c) vulnerable plaques.

**Figure 2:** Experimental setups.

**Figure 3:** Velocity distribution at three positions of phantom plaques with different degrees of stenosis. (a) 30% of stenosis; (b) 50% of stenosis; (c) 70% of stenosis.

**Figure 4:** Comparison of the distribution of special biochemical markers between the two groups of patients. ( ^*∗*^ indicated that the difference was substantial).

**Figure 5:** ROC curves of different risk factors on vulnerable plaques. (a) Age; (b) hyperlipidemia; (c) apoB; (d) ADP; (e) sE-Selection; (f) multiindex combination.

**Figure 6:** AUC values of different risk factors.

**Table 1:** Comparison of baseline data of patients.

Group	Experimental group	Control group	*P*
Age (years)	49.5 ± 9.4	50.8 ± 8.7	0.23
Sex (male/female)	78/24	74/48	0.68
Smoking history (%)	37.3	33.6	0.35
Hyperlipidemia (%)	42.2	40.2	0.74
Family history (%)	8.8	8.2	0.79
Body mass index	25.8 ± 5.1	25.4 ± 4.9	0.81
Framingham score	5.2 ± 2.3	3.1 ± 1.4	0.02

**Table 2:** Comparison of the levels of general biochemical markers in the serum of the two groups of patients.

Related indicators	Experimental group	Control group	*P*
Fasting blood glucose (GLU)	5.44 ± 1.25	5.41 ± 1.08	0.105
Total cholesterol (TC)	4.59 ± 0.87	4.50 ± 1.02	0.096
Triglyceride (TG)	1.74 ± 0.56	1.52 ± 0.47	0.087
High density lipoprotein (HDL-C)	1.05 ± 0.22	1.16 ± 0.33	0.021
Low density lipoprotein (LDL-C)	3.23 ± 1.39	2.96 ± 0.93	0.009
Apolipoprotein A1 (apoA 1)	1.26 ± 0.27	1.25 ± 0.31	0.181
Apolipoprotein B (apoB)	0.98 ± 0.19	0.94 ± 0.24	0.006
apoB/A1	0.75 ± 0.17	0.72 ± 0.17	0.078
Apolipoprotein E (apoE)	4.59 ± 1.51	4.61 ± 1.33	0.123
Creatine kinase (CK)	83.22 ± 11.36	94.18 ± 16.73	0.004
Creatine kinase isoenzyme (CK-MB)	11.25 ± 2.89	11.04 ± 1.73	0.058
Troponin T (CTnT)	0.005 ± 0.001	0.004 ± 0.001	0.339
High-sensitivity C-reactive protein (Hs-CRP)	0.133 ± 0.038	0.139 ± 0.032	0.291

## Data Availability

The data underlying the results presented in the study are available within the manuscript.
